RETRACTED

# Design and Simulation of Logistics Network Model Based on Particle Swarm Optimization Algorithm

**DOI:** 10.1155/2022/1862911

**Published:** 2022-07-08

**Authors:** Lin Tan, Ailing Zhang, Sha Li, Minghua Ding, Pengfei Liu

**Affiliations:** ^1^Shandong Vocational and Technical University of International Studies, Rizhao 276800, China; ^2^Rizhao Economic and Technological Development Zone Economic Development Group Co., LTD, Rizhao 26800, China

## Abstract

With the continuous development of e-commerce, logistics and express services have penetrated into every aspect of people's life. Research on the optimization of logistics network model is helpful to reduce the waste of routes, improve the utilization rate of transportation tools and hubs, and thus reduce the organizational cost of logistics. In this paper, the basic model of hub-and-spoke network (HSN) is constructed based on the principle of minimizing the connection distance and total cost between hubs. By discretizing the particles in the continuous motion space, the discrete particle swarm optimization (PSO) algorithm is designed and the Exchange () exchange function is used to improve its search strategy to update the individual optimal value and the global optimal value. Finally, the improved double-layer discrete PSO algorithm is obtained to solve the logistics network model. The results show that the optimized PSO algorithm has faster convergence speed and higher precision, and the application of the logistics network model is helpful to integrate logistics resources, reduce logistics costs, and improve logistics efficiency.

## 1. Introduction 

With the continuous development of e-commerce, logistics and express services have penetrated into all aspects of people's lives. Since China's accession to the World Trade Organization (WTO), the structure of logistics network has gradually begun to upgrade that many multinational companies have begun to merge and acquire with the help of trade contacts, which make the original independent economy integrate into the global trade environment [1, 2]. As a result, the supply chain network has entered the network planning of China's modern logistics development. With the increase of network scale, network participants have also begun to increase, and the relationship between participants has become more complex [3]. At present, China's modern logistics industry is in the golden period of development, it is necessary to accelerate the development of regional economy in order to meet the market competitiveness of enterprises.

In modern logistics, distribution is an important link directly connected with consumers, and the distribution cost is the highest proportion in the process of logistics service. The high-efficiency service and low cost brought by scientific distribution path planning directly reflect the core competitiveness of enterprises. In China's current logistics management, a reasonable distribution route can not only improve the user experience with higher performance time but also reduce the operating cost of the enterprise by controlling the distribution cost [4, 5]. In the process of one-way logistics distribution, the standard of constructing network optimization model takes the cost of logistics distribution in the network as the goal and takes into account the traffic volume of each station and the capacity limit of transfer hub. In order to optimize the logistics network, we should select the transit hub site to be established among the several alternative hub sites given, so as to optimize the logistics network [6–8]. In addition, some studies have shown that the appropriate hub station is selected as the intermediate exchange station or transfer station among the nodes in the network. The transfer data, mail, express delivery, parcel, cargo, or air passengers from different places are collected on the established hub, and the resources from different sources are combined at the hub and sent to other hubs or final destination nodes, respectively, which is conducive to the formation of a processing center with certain product flow. At the same time, it will form new industrial agglomeration benefits [9, 10].

RETRACTED

At present, there are many optimization methods for logistics network, which are mainly divided into precise method and heuristic algorithm. However, they have some limitations, such as large calculation, large storage, and unreasonable path design, which leads to high cost of logistics distribution. While PSO has the advantages of simple process, convenient implementation, fast training speed, and high-solution quality, which is widely used. However, in practical application, it is easy to produce premature convergence and poor local optimization ability, which cannot meet the current needs of logistics network optimization. In order to overcome the shortcomings of PSO algorithm, this paper designs a different search strategy from the standard PSO algorithm to better solve the logistics network model.

## 2. Design Logistics Network

### 2.1. Analysis of Logistics Service Process

Logistics service transaction process refers to the logistics service information released by logistics service providers and logistics demand information released by customers provided by multilogistics service trading platforms under the complex Internet environment. Then, according to the released information, the supply and demand sides will contact, negotiate, negotiate, and conclude a transaction with the logistics service providers or customers meeting their own needs; finally, the provider completes the logistics service. The traditional logistics service transaction process is shown in Figure 1.

RETRACTED

Customers and logistics service providers can find the corresponding service information through the Internet according to their own needs where customers can obtain the logistics orders of the corresponding providers through the platforms and the providers can also track the corresponding logistics. The payment method between customers and logistics service providers is through the third-party payment platform that can visualize the demand of both sides and optimize the logistics service in this supply chain. The enterprise will show the product information to the customer through the network, the customer through the visitor to visit the website, select the goods to buy, and fill in the order. The manufacturer identifies the customer through the order, informs the charging method, and informs its application system to organize the sourcing process. The customer interacts with the financial department to transfer funds through electronic settlement. The financial department notifies the buyer and seller of the result of the transfer of funds by e-mail (or other means). The factory organizes the goods and delivers them to the customers.

### 2.2. HSN

Logistics network is a kind of practical network form which can meet the demand dispersion and multidirectional logistics activities in order to reduce the organization cost of logistics at the same time, which is also a form of spatial organization with logistics economic activities formed by logistics center city, logistics economic belt, and logistics channel [11].

For a country with a vast territory like China, in order to achieve the goal of maximizing benefits, the HSN can establish connections with the surrounding subnodes in a large range of core areas at a suitable distance, so as to avoid waste due to the establishment of too many hubs and lines, and improve the utilization rate of transportation tools, which is also helpful for different levels of nodes to play their respective roles and improve their economic benefits.

As shown in Figure 2, the 6-node through network is taken as an example; compared with the fully connected network, the HSN has fewer connecting lines and the connection mode between points has also changed. Assuming that from node 1 to node 2, the path in hub spoke network is 1–4–5–2, while in-through network is 1–2. Therefore, there are fewer links in a HSN.

RETRACTED

Based on the above analysis, this paper adopts HSN to establish the basic logistics network structure. In the actual network structure, it mainly involves two layers of HSN, the upper network is the location of hub-level sites, the lower level network is the distribution of sales stores, the connection of the two-tier network and the hub level stations radiate the range of sales stores, the design adopts the double-layer HSN as the main transportation network, and its schematic diagram is shown in Figure 3.

Like other economic network systems, the development of HSN will also be affected by facility operators, users, and network managers. It provides more network services for a wider area by increasing hub points, which can improve the number of direct services between key nodes and provide customers with more frequent transit services [12]. In logistics transportation, it can also bring huge economic advantages to logistics service providers and carriers and reduce the cost caused by inconvenient transportation.

### 2.3. Logistics Network Model

The choice of the number of hubs and the capacity of their respective flows are important constraints to be considered in the design of HSN. The standard of constructing the network optimization model takes the total logistics distribution cost in the network as the goal and takes into account the traffic volume of each station, the capacity limit of the transit hub station, and the selection of the site location to meet the requirements. In order to optimize the network, the transfer hub station to be established is selected from several alternative hub stations. Therefore, in this study, it is assumed that the hub station of logistics distribution should meet the following conditions:

1. Goods from the general warehouse to each sales subnode must be transferred through the transit hub.
2. Each subnode can only transfer through one transit hub, and the transfer form through two or more transfer hubs is not considered.
3. The unit distance from hub transfer center to subnode, unit freight volume, demand of subnode, transfer cost and distribution cost, average transportation cost per unit freight volume are known.
4. There are two routes of HSN goods circulation in this study: general warehouse-subwarehouse-store; general warehouse-subwarehouse-subwarehouse-store. Therefore, unlike the conventional HSN, there is no reverse transportation from the subnode to the hub node.

Therefore, the logistics network model is as follows:

(1) $$\begin{array}{c} \begin{array}{cc} \min, & \sum_{i}\sum_{j}\sum_{k}w_{ij}x_{ij}c_{ij}+\sum_{i}\sum_{j}\sum_{m}w_{ij}x_{jm}c_{jm}+\sum_{i}\sum_{j}\sum_{m}w_{ij}x_{ik}x_{jm}c_{jm}+d\sum_{j}x_{jJ},\\ \text{s.t.}, & \left(n-p+1\right)x_{jj}-\sum_{i\in n}x_{ij}\geq 0,\;j=1,2\ldots ,n, \end{array}\\ \sum_{j\in n}x_{ij}=1,\;\forall i\in n,\\ \sum_{j\in n}x_{jj}=p,\\ x_{ij}=\left\{\begin{array}{cc} 1, & \text{the central hub }i\text{ is established at }j,i\text{ is connected with }j,\\ 0, & \text{other conditions}, \end{array}\right.\\ x_{jj}=\left\{\begin{array}{cc} 1, & j\text{ is the central hub},\\ 0, & \text{other conditions,} \end{array}\right. \end{array}$$

where variable *w*_*ij*_ is the product demand from *i* to *j*, *c*_*ij*_ is the cost required by the transport flow from *i* to *j*, and *d* is the construction cost of the central hub. If *i* is connected to the central hub, *x*_*ij*_ is 1; otherwise, it is 0; if point *j* is the hub, *x*_*ij*_ is 1; otherwise, it is 0.

RETRACTED

## 3. Logistics Network Model Based on PSO Algorithm

### 3.1. PSO Algorithm

The basic PSO algorithm searches in the real continuous space, but in practical engineering applications, the variables to be solved may be discontinuous. Therefore, when solving the problem, this paper designs a discrete PSO algorithm to map the motion space of continuous particles, where the speed of PSO is equal to the value of 0 in the space of PSO, but the value of particle's state space is only 0 or 1, the velocity at each position represents the probability that the particle will take a value of 0 or 1 at that position.

The algorithm starts from the randomly generated initial population and assigns individual optimal position and fitness value to each particle's position and fitness value. According to the individual optimal position and fitness value, the global individual optimal value and fitness value are found [13]. The algorithm flow is shown in Figure 4.

The position of the discrete PSO algorithm are updated as follows:

(2) $$\begin{array}{c} v_{i}^{d}\left(t+1\right)=\omega^{*}v_{i}^{d}\left(t\right)+c_{1}r_{1}\left(t\right)\left[p_{i}^{d}\left(t\right)-x_{i}^{d}\left(t\right)\right]\\ +c_{2}r_{2}\left(t\right)\left[p_{g}^{d}\left(t\right)-x_{i}^{d}\left(t\right)\right]. \end{array}$$

The update mode of speed is shown in

(3) $$\begin{array}{c} s\left(v_{i}^{d}\right)=\frac{1}{1+\text{exp}\left(-v_{i}^{d}\right)}, \end{array}$$

(4) $$\begin{array}{c} x_{i}^{d}=\left\{\begin{array}{cc} 1, & r<s\left(v_{i}^{d}\right),\\ 0, & \text{others,} \end{array}\right. \end{array}$$

where *s*(*v*_*l*_^*d*^) represents the probability that the current particle trajectory is 1 and rand() represents a random number within the range of [0, 1].

When solving the model with the help of discrete particle swarm optimization algorithm, the solution vector in the solution space, namely the particles in the particle swarm, should be coded and designed. Each solution should be regarded as a particle, the dimension of the particle is the number of nodes, and the decision variable *x*_*i*_^*j*^ is in the form of *N* × *D*, where *N* represents the number of particles scattered in the solution space is *N*, and the *N*-th line represents the situation where the establishment of facility point is selected. If the site is selected as the location of establishment of facility, *x*_*i*_^*j*^=1, otherwise *x*_*i*_^*j*^=0. Restricted by constraints, each row has a maximum of *P* facilities, that is, the value of only P location is 1, and the other facilities are all 0. The location of subnodes is divided according to the distance from the established facilities.

RETRACTED

Different from the standard PSO algorithm, the search strategy of the discrete PSO algorithm designed in this paper is as follows:

(5) $$\begin{array}{c} w^{t+1}=w^{t}\cdot \beta ,\\ s_{1}=w^{t}⊗\text{exchange}\left(x_{i}\left(t\right)\right)\\ s_{2}=c_{1}⊗\text{exchange}\left(p{\text{best}}_{i}\left(t\right)\right),\\ s_{3}=c_{2}⊗\text{exchange}\left(g\text{best}\left(t\right)\right),\\ x_{i}\left(t+1\right)=\text{best}\left(s_{1},s_{2},s_{3}\right), \end{array}$$

where *W* represents the location of subnodes and *β* is the iterative coefficient. In each iteration, considering the position vector of each particle, the particles with the current individual optimal value and the global optimal value are updated by using the Exchange (), where each particle generates a random number between 0 and 1 and selects the random number less than the user-defined inertia weight. Exchange () represents the exchange of a randomly selected facility with another randomly selected node, that is to say, nodes with facilities are randomly selected, and the facilities in this node are carried to other randomly selected nodes without facilities.

### 3.2. Model Solution

Based on the analysis of logistics network model, this paper proposes an improved double-layer discrete PSO algorithm to solve the HSN. The upper-hub site selection scheme is used to randomly generate feasible hub sites, and the improved discrete PSO algorithm is used to optimize it, with the help of the lower-level PSO algorithm, the subnode allocation scheme is optimized again, and then through multiple iterations, the approximate optimal solution of the HSN is obtained when the stopping condition of the algorithm is satisfied. The specific steps are as follows:

**Step 1 .**

Given initialization conditions, each particle is a random sequence of 0–1 in *D* dimension and the constraint conditions are checked. Set the population size *N*, the inertia weight *w*, the reduction factor *β*, the values of learning factors *c*_1_ and *c*_2_, and the maximum iteration times *T*.

RETRACTED

**Step 2 .**

Initialize the population of particles and the velocity *V*, that is, define the position and velocity of each particle.

**Step 3 .**

Change the inertia weight in the current iteration number, so as to calculate the corresponding fitness function particles *X* separately is the total cost of the current location scheme, where the cost is the optimal cost value of the optimal subnode layer location division when the current hub site is selected.

**Step 4 .**

*X* is taken as the initial individual optimal value *p*best, and *p*Best with the minimum objective function value is substituted into *g*best as the initial global optimal position.

**Step 5 .**

Adjust the current particle according to a certain probability, and select the optimal solution from *s*_1_, *s*_2_, and *s*_3_ as the updated particle.

**Step 6 .**

Judge whether the end condition is reached (usually to get the best position or reach the preset number of iterations *T*). If the end condition is reached, the algorithm is terminated; otherwise, return to Step 2.

Integer coding is used in the particle coding of both the upper-hub site and the lower-non-hub site. The site selection scheme of hub-and-spoke network is shown in Figure 5.

For the problem of HSN location with *P* = 3, it is assumed that the sequence of {3, 7, 8} is a possible solution set of hub site location. When the exchange function is applied to exchange, two values need to be derived, one is used to determine the hub value to change, and the other is used to update the hub site to the new hub site. Therefore, the selection and optimization of model subnodes are shown in Figure 6.

When the subnode location scheme of the lower layer is divided, its principle is similar to that of the upper layer, but it should be noted that the selection scheme of the hub site must not be changed in the lower layer.

## 4. Simulation and Results

### 4.1. Problem Description

In the two-layer HSN, the nodes of the first layer network are the franchise stores and direct stores of the company, and they are collectively referred to as stores. The operation of the stores is the secondary hub for the distribution, while the nodes of the second layer network are hub-layer sites. In this application, the sample data consists of logistics distribution centers and 14 demand points. In addition, each service area takes city a as the receiving and dispatching center. The coordinate data of the customer node in the example is shown in Table 1.

The parameters used in this study are set as follows: population size = 100, learning factors *c*_1_ and *c*_2_ are both 2, inertia weight *w* = 0.9, maximum iteration times maxgen = 500, calculation times Time = 10, dimension *D* = number of hub stations + number of vehicles −1, and learning period *T* is set to 50.

RETRACTED

### 4.2. Results and Discussion

#### 4.2.1. Analysis of Model Effectiveness

Matlab is used to run the algorithm to get the shortest distance. The variation of fitness value of the optimal particle in the iteration process of standard PSO algorithm and optimized PSO algorithm is shown in Figure 7.

The PSO algorithm showed precocious convergence when it evolved to the 23rd generation. In the 210th generation, it seldom improved but fell into the second local optimal. It did not improve again until the 235th generation, and the optimal solution that could be found was only 260. While the optimized algorithm found the optimal result of 330.55 in the 35th generation. Because of the application of self-correcting strategy, it ensured the regularity of the correct running direction of particles in the early stage, reduced the waste of time and resources brought by the incorrect guidance of particles, and thus achieved faster convergence. At the same time, it is easy to see that due to the use of exchange strategy, the optimized algorithm has more obvious advantages in solving 14 customer point problems. The dimension of population particles increases with the increase of the number of customers, which make the solution more difficult, while in this paper, by improving the exchange strategy of overall evaluation method, the problem of interdimension interference is effectively avoided, and the high-precision solution ability of exchange strategy is brought into play.

The logistics network distribution path based on discrete PSO is shown in Figure 8.

According to Figure 8, the shortest path optimized by the logistics network model proposed in this paper is 203 km, which is 67 km less than the previous transportation route (the total length is 270 km). Distribution distance of the optimal path is reduced by 24.8% compared with the traditional transportation route before, whose optimization effect is obvious.

#### 4.2.2. Supply Chain Optimization Scheme

In the existing hub network, hub sites are selected as candidate sites for analysis, and the service level of the existing hub network is reduced or improved. The optimization strategy of logistics company's supply chain is as follows:

1. Optimize the number of secondary hub sites, reduce the operating costs of hub sites, and improve the utilization of each hub site.
2. According to the situation of the total warehouse and transportation hub, the transportation cost of the second-level transportation hub should be optimized according to the different situation of the transportation hub.
3. Optimize the radiation range of secondary hub stations to make the distance between each store and secondary hub station the shortest, and reduce the transportation time.

RETRACTED

The total cost variation of network location is shown in Figure 9.

As can be seen from the figure, the cost of delivering products from hub sites to its stores is still high. The total logistics cost is 9,76,400 yuan. When 16 distribution centers are established and other assumptions are met, the total cost is 3,75,800 yuan. However, if the number of hub sites continues to increase, the cost will start to increase gradually.

## 5. Conclusion

In this paper, by discretizing the motion space of continuous particles and adopting the search strategy based on exchange function, a hub-and-spoke logistics network model based on double-layer PSO algorithm is proposed. The upper layer of the model selects the hub site scheme, and the lower layer optimizes the distribution scheme of the subnodes. The simulation results show that, the optimized PSO algorithm has faster convergence speed and higher precision. The results of case analysis show that the distribution distance of the optimal path solved by the logistics network model designed in this paper is 24.8% less than the traditional transportation distance before. When the number of hub stations is 16, the total logistics cost is the lowest, which is 3,75,800 yuan. To sum up, the model constructed is helpful to integrate logistics resources, reduce logistics costs, and improve logistics efficiency.

## Figures and Tables

**Figure 1:** Traditional logistics service process.

**Figure 2:** Comparison of different network structures.

**Figure 3:** Structure of the double-layer logistics network structure.

**Figure 4:** PSO algorithm flow.

**Figure 5:** Example of the logistics network location scheme.

**Figure 6:** Optimization of logistics network nodes.

**Figure 7:** Fitness values of optimal particles in different algorithms.

**Figure 8:** The optimal path based on the logistics network model.

**Figure 9:** Total cost of network location.

**Table 1:** Node coordinate.

Node	*X* coordinate	*Y* coordinate
A	37	52
B	49	49
C	52	64
D	20	26
E	40	30
F	21	47
G	17	63
H	31	62
I	52	33
J	51	21
K	40	40
L	35	45
M	60	64
N	65	35

## Data Availability

The dataset can be accessed upon request to the corresponding author.
